# A Real-Time Clinical Decision Support System, for Mild Cognitive Impairment Detection, Based on a Hybrid Neural Architecture

**DOI:** 10.1155/2021/5545297

**Published:** 2021-06-21

**Authors:** Carmen Paz Suárez-Araujo, Patricio García Báez, Ylermi Cabrera-León, Ales Prochazka, Norberto Rodríguez Espinosa, Carlos Fernández Viadero, for the Alzheimer's Disease Neuroimaging Initiative

**Affiliations:** ^1^Instituto Universitario de Ciencias y Tecnologías Cibernéticas, Universidad de Las Palmas de Gran Canaria, Las Palmas de Gran Canaria, Spain; ^2^Departamento de Ingeniería Informática y de Sistemas, Universidad de La Laguna, La Laguna, Spain; ^3^Czech Institute of Informatics, Robotics and Cybernetics, Czech Technical University, Prague, Czech Republic; ^4^Department of Computing and Control Engineering, University of Chemistry and Technology, Prague, Czech Republic; ^5^Unidad de Neurología de la Conducta y Memoria, Hospital Universitario Nuestra Señora de Candelaria, Santa Cruz de Tenerife, Spain; ^6^Servicio de Psiquiatría, Hospital Universitario Marqués de Valdecilla, Santander, Spain; ^7^Center for Imaging of Neurodegenerative Disease San Francisco VA Medical Center University of California, San Francisco, USA

## Abstract

Clinical procedure for mild cognitive impairment (MCI) is mainly based on clinical records and short cognitive tests. However, low suspicion and difficulties in understanding test cut-offs make diagnostic accuracy being low, particularly in primary care. Artificial neural networks (ANNs) are suitable to design computed aided diagnostic systems because of their features of generating relationships between variables and their learning capability. The main aim pursued in that work is to explore the ability of a hybrid ANN-based system in order to provide a tool to assist in the clinical decision-making that facilitates a reliable MCI estimate. The model is designed to work with variables usually available in primary care, including Minimental Status Examination (MMSE), Functional Assessment Questionnaire (FAQ), Geriatric Depression Scale (GDS), age, and years of education. It will be useful in any clinical setting. Other important goal of our study is to compare the diagnostic rendering of ANN-based system and clinical physicians. A sample of 128 MCI subjects and 203 controls was selected from the Alzheimer's Disease Neuroimaging Initiative (ADNI). The ANN-based system found the optimal variable combination, being AUC, sensitivity, specificity, and clinical utility index (CUI) calculated. The ANN results were compared with those from medical experts which include two family physicians, a neurologist, and a geriatrician. The optimal ANN model reached an AUC of 95.2%, with a sensitivity of 90.0% and a specificity of 84.78% and was based on MMSE, FAQ, and age inputs. As a whole, physician performance achieved a sensitivity of 46.66% and a specificity of 91.3%. CUIs were also better for the ANN model. The proposed ANN system reaches excellent diagnostic accuracy although it is based only on common clinical tests. These results suggest that the system is especially suitable for primary care implementation, aiding physicians work with cognitive impairment suspicions.

## 1. Introduction

The rising trend of an aging population is an enormous social and economic challenge because of the high prevalence of noncommunicable diseases [1]. Dementia, with Alzheimer disease (AD) as its main cause, and cognitive impairment (CI) are a public healthcare challenge.

The MCI concept was proposed to group patients that only display intermediate cognitive deficit between normal aging and the dementia stage, without significant functional impact [2]. These patients present an increased risk of conversion to dementia, with annual rates between 5 and 10% [3]. This figure targets that population as a key objective for early detection and the introduction of measures that could delay its advancement. Early detection of MCI is also considered beneficial because it allows for treatment in the initial stages, which can extend the autonomy of the patients and reduce uncertainty for the family and the patient. Authors in this field have made recommendations for future research that focuses on the use and development of appropriate functional and neuropsychological measures and combinations of them which will improve diagnostic accuracy [4].

Diagnostic procedure for CI is usually initiated by general practitioners. The level of detection at primary care setting is still low, in particular for MCI [5]. Diagnostic protocols are based mainly on clinical records and short cognitive tests, but barriers such as low suspicion index or difficulties about understanding cut-offs have led to low levels of diagnostic accuracy. Furthermore, in CI, the evolution from healthy aging to AD, through the MCI, does not precisely fit a linear model [6], leaving a rather complex problem with nonlinear characteristics. To solve these drawbacks, an approximation based on neural computation for detection of MCI is proposed.

Artificial neural networks can be defined as a cognitive information processing structure (massively parallel dynamical system) based upon models of brain function which are intended to interact with the environment. They are composed of highly interconnected computational elements with a graph topology. Its most appealing property is its learning capability. The ANN behavior emerges from structural changes driven by local learning rules, and they are capable of generalization. They can capture high-dimensional inputs and generate relationships between the inputs and outputs from a training set. In addition, this data-driven procedure also captures the similarity in the input that results in generalizations. They can approximate any real valued function mapping and face tasks close to processes which are thought to occur in the brain.

ANNs can be characterized in the three following levels: connectivity topology, neurodynamics, and learning. Connectivity topology indicates the shape in which the different neural processing elements are interconnected among themselves [7]. Neurodynamics cover the local information processing carried out by the units [7]. Learning is the capacity of a system of absorbing information from the environment, without a need for the system to be programmed externally. The learning processes produce changes in the network in order to try and achieve a new way to respond more efficiently to the specific task.

Multiple computational and mathematical methods have been proposed in the diagnosis of dementia [7, 8], creating an interesting scientific field where a wide body of work exists. In general, the majority of developed research is centered on the detection of the existence or absence of a dementia, usually AD, or performs a differential diagnosis between two types of dementia, or a diagnosis between AD and MCI [9–11], or in longitudinal studies, the identification of conversion from MCI to AD [12, 13].

In this paper, we introduce a different and innovative proposal, which is directed towards perhaps the most effective point of intervention, namely, the estimate of MCI. The main contributions of our proposal are the following: using ANNs, we provide a tool to assist in the clinical decision-making that facilitates a reliable MCI estimate, with simple and multimodal diagnostic criteria. It is useful in any clinical setting but specially in primary care. Our model provides performance levels greater than those normally obtained with clinical and/or computational methods. These levels are also above the threshold of diagnostic precision that is recommended as optimal to consider a biological test such as an AD biomarker [4, 14].

The primary aim of this work is to explore the ability of a hybrid ANN-based system to differentiate healthy controls and MCI patients. A secondary objective is to compare the ANN-based system and physician's clinical diagnostic.

## 2. Materials and Methods

### 2.1. Data Set and Feature Selection

Data used in the preparation of this article were obtained from the Alzheimer's disease Neuroimaging Initiative (ADNI) database (http://adni.loni.usc.edu). The ADNI was launched in 2003 as a public-private partnership, led by Principal Investigator Michael W. Weiner, MD. The primary goal of ADNI has been to test whether serial magnetic resonance imaging (MRI), positron emission tomography (PET), other biological markers, and clinical and neuropsychological assessment can be combined to measure the progression of mild cognitive impairment and early Alzheimer's disease. ADNI is also a comprehensive study of imaging and omics in AD [15].

The ADNI database includes different diagnostic groups of AD and MCI. Criteria for subject selection are given in ADNI protocol. Our dataset includes the scores of three commonly used neuropsychological tests along with the years of education and age, relative to 203 normal control subjects and 128 subjects who revealed a MCI. The diagnostic instruments, essentially dedicated to the cognitive and functional assessment, are the MMSE [16], the FAQ [17], and GDS [7].

Table 1 depicts some information about the demographic features, test results, and education level of the subjects. The data set was split up in two parts: a training set with 255 persons and a test set with 76. Both have similar statistical characteristics, and they are balanced in the MCI subjects and normal control subject ratio.

We propose the design of a system that efficiently, simply, and quickly detects MCI, using only a set of reduced clinical criteria commonly used in primary care. This aim is achieved by joining a simple and powerful feature selection scheme, the wrapper method [18] with the neural computing methodology. This method uses an ANN as a fitness function and searches for the best subset of features in the feature space. The wrapper methodology offers a simple but powerful way to address the problem of feature selection, even though it is computationally more complex and requires more execution time than other feature selection methods. A backward elimination search strategy has been applied, with two restrictions: the minimum dimension of the input vector must be two, and all the input vectors must have at least one diagnosis criteria. A total of 24 different feature vectors were obtained. This method is used because of its simplicity and its universal use, and the generated space of all possible feature subsets under development is not too large; thus, the search is not computationally hard.

### 2.2. Counterpropagation Network

The foundation of modular neural networks (MNN) relies on the possibility that a single neural network can be freely combined with other types of artificial neural networks. Each monolithic neural network can be considered as a module. An important aspect of the MNN is its biological background, as biological neural systems also are characterized by a combination of a hierarchy of networks. Modular neural networks are generally more powerful than flat unstructured ones [19]. The key idea in these networks is to solve complex problems in a simpler, quicker, and more manageable way [20]. One of these highly effective modular networks is Counterpropagation Network (CPN) [21, 22].

The Counterpropagation Network (CPN) is a hybrid modular neural network [21]. It is seen as an extension of the Kohonen approximation and is made up of a network hierarchy, each one specialized in different tasks, by using similarities with natural systems. CPN faces the classification process in a modular way using different learning algorithms. One part of the network uses self-organizing learning for quantification which processes initial input, and afterwards, a supervised learning scheme occurs, which deals with the discrimination process performed by the network [20].

Therefore, CPN is a modular neural architecture of two independent-learning cascaded layers (Figure 1). The first layer is competitive, the Kohonen self-organizing Map (SOM). It produces a clustering of the input space, preserving its topology, which is related to an *n*-dimension Voronoi diagram and maps to a space with a reduced dimensionality, generally two. SOM presents an input layer that has a full-connectivity with the output layer by means of excitatory connections. The output layer is organized in an *m*-dimensional space which matches the desired map form. This output layer is characterized by a neighborhood relationship that is present between the nodes, typically from a square or hexagonal lattice shape or another geometric shape. This layer may even have a thyroidal connectivity structure. All of the units in this layer simultaneously present inhibitory lateral connections among neural neighbors as well as excitatory self-connections. Said connections are those that facilitate the competitive process while searching for the winning neuron. Its neurodynamics in practice are usually simplified by carrying out the Euclidean distance of the inputs and the neuron prototypes (Equation (1) and Equation (2)). The winning unit is the one which is closest (higher similarity) to the input vector.

(1) $$\begin{array}{c} {\text{net}}_{l}\left(x\right)=\left\|x-w_{l}\right\|, \end{array}$$

(2) $$\begin{array}{c} u_{l}=\left\{\begin{array}{cc} 1 & \text{if }l=\arg\underset{k}{\min}\left({\text{net}}_{k}\left(x\right)\right),\\ 0 & \text{otherwise}. \end{array}\right\} \end{array}$$

The unsupervised learning process belongs to the winner take all category, similar to the simple competitive learning process. The main variations are seen in the modification of the synaptic weights, which not only affects the winning neuron but also to a lesser degree the set of neurons in the winner's neighborhood *N*, and consequently are able to generate topological relations (Equation (3)).

(3) $$\begin{array}{c} \Delta w_{li}=\left\{\begin{array}{cc} \alpha \left(x_{i}-w_{li}\right) & \text{if }l\in N\left(\arg\underset{k}{\min}\left({\text{net}}_{k}\left(x\right)\right)\right),\\ 0 & \text{otherwise}. \end{array}\right\} \end{array}$$

An interesting aspect of this neural architecture lies in the neighborhood relationship between nodes, and the learning rates are functions of time. They decrease during the training period.

The Grossberg layer carries out the second stage of the CPN. Its neurodynamic is given by a linear combination of the SOM output. Each unit on this layer rapidly reaches an equilibrium value equal to the value of the actual weight in the connection to the winning unit of the competitive layer, following (Equation (4)).

(4) $$\begin{array}{c} y_{j}=\underset{l}{\sum }u_{l}z_{jl}, \end{array}$$

A threshold on these output units can be established in classification processes. When the activation value of the unit is greater than the threshold, the input pattern is considered to belong to the class, which is represented by that unit. Management of this threshold allows the network to be tuned, resulting in classifiers with different sensitivities or specificities.

This layer uses *outstar* learning [23]. A straightforward gradient descent on this cost function provides the necessary weight update (Equation (5))

(5) $$\begin{array}{c} \Delta z_{jl}=\gamma \left(d_{j}-y_{j}\right)u_{l},, \end{array}$$

where *d*_*j*_ is the value of the wanted output for the *j* neuron and *γ* is the learning rate.

The advantages obtained with this model mainly lie in the reduction of complexity regarding equivalent monolithic models, allowing for simultaneous training of both layers, increasing strength and the incremental character of generated applications, and its rate in computing time. The increase in the computing rate is achieved because of the simplification in the self-organizing stage [20].

Different configurations of CPNs, for all 24 corresponding feature vector, were developed by varying their parameters. Hexagonal and square neighborhoods in SOM, with toroidal and/or planar connectivity structure, were used. The threshold value of the Grossberg layer is chosen in such a way that the values of sensitivity and specificity for each network are the most similar possible. The CPN input space was normalized and scaled into linear format.

### 2.3. Performance Measures

The efficacy of the proposed diagnostic system is determined using different performance measures: sensitivity, specificity, accuracy, the receiver operating characteristic (ROC) curves, and the area under the ROC (AUC).

Errors made by a classifier in a specific scope, such as the medical setting, can lead to a different level of importance. Two measures, sensitivity and specificity, are commonly used to consider this difference in the importance of the diagnosis. Sensitivity is the probability that a test result will be positive when the disease is present (true positive rate (TPR)), and specificity is the probability that a test result will be negative in the absence of the disease (true negative rate (TNR)). In the context of binary classifiers, these measures are equivalent to calculating accuracy.

Another aspect that should be borne in mind when comparing classifiers or when their performance is analyzed is the precision of the classifiers on the parameter adjustment, since they influence detected TPR and TNR. The use of ROC curves [24] is a good method for this evaluation. ROC is a bidimensional graphical representation of sensitivity versus (1 − specificity) according to how the classifier discrimination threshold changes. Threshold in this work refers to Grossberg layer of CPN. AUC is a very good measure of fit for classifiers and is used in this work. AUC is statistically consistent and more discriminating measure than accuracy [25].

In order to evaluate the clinical value of our proposal with regard to the simultaneous utilization of cognitive and functional measures, the clinical utility index (CUI) [26] and the corresponding optimum cut-off over each one of the FAQ, MMSE, and GDS tests were also used. In this way, we have deemed the clinical applicability of the diagnostic system, in the same sense as the clinical applicability of a test [27].

In order to define a clinically valuable diagnostic test or diagnostic system, high values of positive predictive value and high sensitivity values are needed. In a formal way, the positive utility index (for rule-in accuracy) is a product of sensitivity and positive predictive value, and the negative utility index (for rule-out accuracy) is a product of specificity and negative predictive value. Qualitative grades of CUI (CUI+ and CUI-) have been proposed, adapted from *kappa agreement* [26, 27] giving a scores conversion into qualitative grades as follows: excellent utility ≥ 0.81, good utility ≥ 0.64, satisfactory utility ≥ 0.49, and poor utility <0.49 [28].

Lastly, we have also compared the proposed method to reach a reliable and quick diagnosis of MCI, with physicians' performances. Specifically, a neurologist, a geriatrician, and two primary care physicians were involved. All the physicians are blinded with respect to patients, and their diagnoses are only based on the ADNI scales scores, exactly the same data as the hybrid ANN.

## 3. Results and Discussion

Obtained results presented in this section show the efficacy of the proposed diagnostic system.  Table 2 displays the results of the CPN configurations by applying a wrapper method, ordered from highest AUC value of convex ROCs. The optimal CPN configuration occurred with the MMSE, FAQ, and age input combination, reaching 95.11% of AUC, while the same combination, but without age, is slightly worse, AUC of 94.2%. This result is better than that communicated by MMSE and FAQ in the bibliography [26, 29]. The optimal combination is above the threshold of recommended diagnostic precision level for a biological test to be considered as a biomarker of AD [14]. The CUI values for the best CPN configuration were in the range of good clinical utility (CUI + = 0.7147; CUI − = 0.7873) as measured on the Mitchell scale, which confirm the goodness of this proposal.

As seen in Table 2, the best combinations generally included FAQ. This could seem paradoxical when considering that the preservation of daily routines is one of the criteria in the accepted definition of MCI. Nevertheless, ADNI database may have overdimensioned the degree in which the functional level has been affected, and its impact must be considered. GDS was the input variable which contributed the least amount of information when identifying the MCI.

The corresponding optimum cut-off over each of the FAQ, MMSE, and GDS tests was also calculated. These cut-offs allowed us to evaluate the efficacy of individual diagnostic instruments against our proposal, with simultaneous utilization of cognitive and functional measures. As shown in Table 3, their values are worse than the ones produced by the CPN-based system, which combines two of these diagnostic criteria and also considers the risk factor of age. These results can also be observed in the ROC curves for the cut-off of the different scales (Figure 2) and in the convex ROC curves of the two best CPN-based diagnosis systems (Figure 3). The optimal points and the results of the medical experts are indicated on the curves according to Table 2. It is clear that the CPNs are clearly superior to the cut-off points of the tests, outperforming them by more than 6%, with respect to the best of the cut-off point cases and by almost 39% with respect to the worst, considering the AUC value. Regarding sensitivity, the CPN-based system is also better, 6.33% above the sensitivity of FAQ, 10% of the MMSE, and 66.67% above that of the GDS. Similarly, the CPN system shows a better CUI than the one corresponding to each test individually. FAQ was the only measure that reached a CUI+ of good level, -0.6944 (Table 3).

Lastly, as shown in Table 3, the CPN system outperformed clinician results. The best sensitivity was achieved by neurologist, 86.7%, and the best specificity and accuracy were by geriatrician, 93.48% and 78.95%, respectively. On the other hand, primary physicians achieved the lowest sensitivity and specificity values. These results could be explained by the prevalence of MCI, which is much greater in the neurology consultations than in geriatric ones or in primary care. All the physicians' CUIs were also worse than the CPN system. The better results from our system are also noteworthy [30, 31]. This occurs even though our model was simpler and uses less invasive critical criteria, at a cheaper costs and with possibilities of use in all clinical scopes, primary and specialized care.

## 4. Conclusions

We have got all proposed aims, and important conclusions have also reached, in this work. We designed an intelligent system, based on hybrid ANNs, providing a tool to aid in a reliable detection of MCI, which is underdiagnosed, in a primary care setting. It was built on the evaluation of the cognitive and functional domains, considering age and academic studies as modifying factors.

The combination of MMSE, FAQ, and age led to the best diagnostic performance [32]. The proposed CPN system improves the results obtained by statistical methods of other authors. Our method offers greater control when searching for a balance between sensitivity and specificity. It works with the simultaneous use of multimodal diagnostic criteria, confirming a higher effectiveness than each separate test. Our proposal overcomes methodological challenges, such as the choice of an administration strategy and the calculation of cut-offs, which are present when multiple tests are used. It provides evidence that age was more significant than academic studies for an improvement in the detection of MCI. The CPN diagnosis system performances were not impeded by physician bias, which offers greater reliability.

We propose, based on the obtained results from our study, that the best solution to solve MCI detection in a primary care setting and in the general consultations of neurology and geriatrics could be to use systems incorporating diagnostic aid based on hybrid ANNs. The use of systems goes beyond the use of cut-offs over different cognitive tests. Under this proposed scenario, it is possible to standardize diagnostic criteria for the detection of MCI, which at present is absent in MCI diagnosis as well as in AD. This tool can also contribute to standardize diagnostic procedures, speeding up the time in consultation and reducing the degree of uncertainty in diagnosis, which are some of the limitations that block the diagnostic work of primary care doctors. Thus, this tool can be specifically appropriate in primary care, which is where the patient enters into the majority of health public systems. It can also be used for the screening and early diagnosis of cognitive impairment. The use of this tool in the diagnosis of MCI is part of the expansion of the e-Health era.

Our study reveals that the use of computational intelligence methods in the design of clinical decision systems for diagnostic aid in the setting of cognitive impairment and dementia is beneficial. These results are very promising and encourage us to continue research along this line. Similar to what occurs in clinical practice, the use of longitudinal information from different visits can be integrated into the ANNs improving precision and reliability of the computational models, so we propose to improve our advances by introducing longitudinal design and extending it into the bimodal diagnostic to the differential, where AD is present. The research is of particular interest given that the moment in which the MCI is diagnosed may be the most effective point for intervention and of significant use for public health planning. This early diagnosis can lead to a delayed progression from the preclinical stage of dementia to the full-blown clinical syndrome.

## Figures and Tables

**Figure 1:** Structure of a Counterpropagation Network.

**Figure 2:** ROC curves for the test set and cut-off points in the different tests.

**Figure 3:** ROC curves for the test set and best CPN system.

**Table 1:** Characteristics of the subjects: demographic features, education level, and test results of the subjects. SD: standard deviation; YOE: years of education.

	Controls	MCI	Total
Subjects	203	128	331
Age mean (SD)	74.1 (6.3)	74.9 (7.2)	74.4 (6.7)
Age range	56.3-89.1	56.3-88.0	56.3-89.1
YOE mean (SD)	16.5 (2.6)	15.5 (3.2)	16.1 (2.9)
YOE range	10-20	4-20	4-20
MMSE mean (SD)	29.1 (1.2)	27.2 (1.7)	28.3 (1.7)
MMSE range	24-30	24-30	24-30
FAQ mean (SD)	0.2 (0.6)	3.6 (4.4)	1.5 (3.3)
FAQ range	0-5	0-20	0-20
GDS mean (SD)	0.8 (1.2)	1.6 (1.5)	1.1 (1.3)
GDS range	0-6	0-5	0-6

**Table 2:** Results for the CPN systems using different input combinations from wrapper method. AUC: area under the ROC; Acc: accuracy; Sen: sensitivity; Spc: specificity; YOE: years of education.

	AUC (%)	Acc (%)	Sen (%)	Spc (%)
Age + MMSE + FAQ	**95.11**	86.84	90.00	84.78
MMSE + FAQ	94.42	85.53	90.00	82.61
Age + MMSE + FAQ + GDS	92.97	**88.16**	86.67	89.13
Age + FAQ	92.25	82.90	96.67	73.91
MMSE + FAQ + GDS	90.98	81.58	86.67	78.26
MMSE + FAQ + GDS + YOE	90.87	86.84	80.00	91.30
Age + MMSE + FAQ + YOE	90.22	86.84	70.00	97.83
FAQ + GDS	90.22	84.21	73.33	91.30
Age + FAQ + GDS	88.44	81.58	86.67	78.26
Age + MMSE + FAQ + GDS + YOE	87.97	**88.16**	80.00	93.48
MMSE + FAQ + YOE	87.75	82.90	70.00	91.30
FAQ + YOE	86.70	85.53	80.00	89.13
MMSE + GDS + YOE	86.49	80.26	73.33	84.78
Age + MMSE + GDS	86.23	84.21	80.00	86.96
Age + MMSE	86.23	80.26	70.00	86.96
Age + MMSE + YOE	86.09	80.26	70.00	86.96
Age + MMSE + GDS + YOE	85.58	78.95	76.67	80.44
MMSE + GDS	85.36	73.68	93.33	60.87
MMSE + YOE	84.31	75.00	93.33	63.04
Age + FAQ + YOE	82.17	81.58	70.00	89.13
FAQ + GDS + YOE	80.58	73.68	83.33	67.39
Age + FAQ + GDS + YOE	80.00	80.26	60.00	93.48
Age + GDS	71.92	65.79	76.67	58.70
Age + GDS + YOE	66.88	60.53	83.33	45.65
Age + YOE	65.69	65.79	56.67	71.74
GDS + YOE	63.41	53.95	90.00	30.44

**Table 3:** Comparison of the results of the optimal CPN system versus cut-off points for the scales and medical experts from the specialized area physicians (neurologist and geriatrician) and the primary care physicians. AUC: area under the ROC; Acc: accuracy; Sen: sensitivity; Spc: specificity; PCP1 and PCP2: primary care physicians.

	AUC (%)	Cut-off	Acc (%)	Sen (%)	Spc (%)	CUI+	CUI-
Optimal CPN system	**95.11**	—	**86.84**	90.00	84.78	0.7147	0.7873
FAQ cut-off	88.80	0/1	**86.84**	83.33	89.13	0.6944	0.7944
MMSE cut-off	80.65	28/29	73.68	80.00	69.57	0.5053	0.5858
GDS cut-off	56.12	2/3	64.47	23.33	91.30	0.1485	0.5900
Neurologist	—	—	77.63	86.67	71.74	0.5778	0.6398
Geriatrician	—	—	78.95	56.67	93.48	0.4817	0.7178
PCP1	—	—	69.74	23.33	100.00	0.2333	0.6667
PCP2	—	—	68.42	20.00	100.00	0.2000	0.6571

## Data Availability

Data used in the preparation of this article were obtained from the ADNI database (http://loni.ucla.edu/ADNI). As such, the investigators within ADNI contributed to the design and implementation of ADNI and/or provided data but did not participate in analysis or writing of this report. A complete listing of the ADNI investigators is available at http://loni.ucla.edu/ADNI/Collaboration/ADNI\_Authorship_list.pdf.
